# Implementation of Evidence in Preventing Postoperative Sore Throat of Patients Undergoing General Anesthesia Intubation Using the i-PARIHS Framework

This article has been retracted.

**DOI:** 10.1155/2022/3151423

**Published:** 2022-07-05

**Authors:** Qian Liu, Yiting Wang, Ruo Zhuang, Lei Bao, Liqun Zhu, Yingfeng Zhou

**Affiliations:** ^1^Anesthesia Operating Room, Affiliated Hospital of Jiangsu University, Zhenjiang City, China; ^2^Evidence-Based Nursing Cooperation Center of Fudan University, School of Nursing, Fudan University, Shanghai, China

## Abstract

**Objective:**

The aim of the study was to assess the effectiveness of the implementation of the best evidence in preventing postoperative sore throat in patients undergoing general anesthesia intubation.

**Methods:**

The related topics of the postoperative sore throat of patients undergoing general anesthesia intubation were systematically searched in the database and evaluated using the Integrated Promoting Action on Research Implementation in Health Services (i-PARIHS) framework. Combined with clinical needs and evidence-based professional judgment, 20 pieces of evidence and 6 examination standards on the management process and evidence implementation plan for the prevention of postoperative sore throat in patients with general anesthesia intubation are summarized, implementing the best evidence into clinical practice in anesthesiology, general surgery, orthopedics, thoracic surgery, and gynecology.

**Results:**

Nurses' knowledge scores and evidence compliance significantly improved after the implementation of the best evidence (*P* < 0.05); the incidence of the postoperative sore throat in patients undergoing general anesthesia intubation decreased from 41.7% to 28.1%.

**Conclusion:**

The i-PARIHS framework effectively prevents postoperative sore throat in patients, providing an effective case for translating evidence into practice based on the i-PARIHS framework.

## 1. Introduction

Postoperative sore throat (POST) is the nociceptive pain caused by the throat and tracheal mucosa injury during tracheal intubation under general anesthesia. The main clinical manifestations are postoperative sore throat, local congestion, and redness, accompanied by hoarseness, low voice, and cough. It will affect eating or even cause fatal injury in severe cases [1]. It has been reported that the incidence of postoperative pharyngolaryngitis and hoarseness is as high as 6.9%∼90.0% [2–4], which causes pain, aggravates patients' difficulty in swallowing and speaking, reduces postoperative comfort, and prolongs patients' hospital stay [5–7]. Therefore, the effective control of POST has great significance in improving the management quality of general anesthesia intubation and the safety of patients. However, there is a lack of clinical practice guidelines and systematic intervention for POST prevention in China, and most measures taken by nurses in a clinic are based on experience and routine. Therefore, this study aims to explore the best evidence for postoperative sore throat prevention in patients with general anesthesia intubation and to conduct clinical translation and implementation to address postoperative sore throat and thus improve the quality of care.

## 2. Methods

### 2.1. Setting and Participants

This study uses the i-PARIHS framework and adopts a controlled before-and-after study. Clinical research was carried out in the anesthesia department, general surgery department, orthopedics department, thoracic surgery department, and gynecology department of a third-class hospital from June 2019 to June 2021, including baseline review before evidence implementation, practice reform, and effect evaluation after evidence implementation.

Five wards in the Affiliated Hospital of Jiangsu University were selected. 151 patients with general anesthesia intubation, patients, and 140 clinical medical staff were included as research objects before and after the implementation of evidence.

The inclusion criteria for patients are as follows: (1) adult (age ≥18 years old); (2) patients undergoing elective general anesthesia; (3) no other underlying medical conditions; (4) patients have no contraindications to anesthesia.

The exclusion criteria for patients are as follows: (1) patients who suspend surgery for some reason; (2) patients who subjectively refuse to participate in the study; (3) patients who objectively cannot cooperate due to mental and audio-visual disorders; (4) patients who lacked complete medical record data; (5) patients who withdraw halfway through the course of treatment. The inclusion criteria for nurses are working for more than 6 months and obtaining a nurse practice certificate; the exclusion criteria for nurses do not agree to participate in the study.

### 2.2. Baseline Survey

#### 2.2.1. Team Formation

Evidence-based expert team and evidence review team include (1) establishment of a review team which consists of 10 members, including one head nurse of the anesthesiology department as the team leader, who plans the overall project and trains the team members to ensure the implementation of evidence transformation. One nursing department director ensures project resources; one teaching secretary is responsible for process decision-making and departmental consultation. Six head nurses and directors are responsible for project support and coordination; one graduate student is responsible for data collection and analysis. (2) There are two members in the evidence-based expert group, including one deputy head of the evidence-based committee who is responsible for the project quality control and guiding the practice plan. A tutor from the Evidence-based Center of Fudan University Nursing tracked, guided, and reviewed the whole project.

#### 2.2.2. Determination of Review Indicators and Review Methods

In addition to the 12 members of the project team, two anesthesiologists from our hospital were invited to evaluate the best evidence of integration in four dimensions, namely, feasibility, suitability, clinical significance, and effectiveness according to the FAME principle.

Combined with the clinical environment of evidence transformation and the resources of our hospital, we turn the items related to the best evidence for clinical implementation into 16 quality inspection indicators (please refer to the Summary of the Best Evidence for Prevention of Throat Pain after General Anesthesia and Tracheal Intubation in the journal of nursing science in 2021 for specific evidence items) and determine the inspection objects and methods of the inspection indicators one by one, as shown in Table 1.

#### 2.2.3. Evaluation Index

(1) Incidence of postoperative sore throat (%) and (2) severity of postoperative sore throat (using Prince-Henry sore throat score [8]) are divided into four grades: no pain feeling when coughing is 0 point; occasionally, there is a pain when coughing, but the absence of pain during deep breathing is 1 point; pain occurs during deep breathing, and it is relieved when quiet is 2 points; there is pain feeling in a quiet state, but within the tolerable range, it is 3 points; when in a quiet state, the pain is severe and unbearable is 4 points. (3) The time at which the patient eats after surgery, (4) the amount of food for patients after the operation, (5) the degree and level of dysphagia were recorded, and Wada test was put forward by Japanese scholar Toshio Wada in 1982 [9], which is the most classic method of swallowing function screening. Washi's drinking water experiment is as follows: patients sit flat and fill a cup of warm water (capacity 30 ml), so that the patient can drink it in a normal state. Carefully observe the patient's drinking process and make records to realize the swallowing function of the patient during this process.

*(1) The Evaluation of the Grade*. Scoring criteria are as follows: 1. Grade I: the patient drank it all at once, and there was no abnormality; 2. Grade II: the time is 0∼5 s, and there was no bucking after drinking twice; 3. Grade III: there is bucking, and the time is 5∼10 s after drinking once; 4. Grade IV: the cough is mild, and the time is 5∼10 s after drinking many times; 5. Grade V: frequent bucking, difficulty in drinking water, time >10 s; (6) comfort (VAS score [10]) was evaluated when the patient was awake. Scoring criteria are a s follows: the feeling of no pain at the wound is 0 points; slight pain in the wound is 1∼2 points; the pain in the wound was slightly obvious, and the number of times of pain was 3∼ points. The pain in the wound is obvious, but within the tolerable range, it is 5∼7 points; the acute pain in the wound cannot be tolerated for 8∼10 points; and (7) investigation and analysis of the mastery of the knowledge (knowledge, attitude, practice KAP).

### 2.3. i-PARIHS

Evidence-based practice model was used to analyze the obstacle factors of clinical transformation of evidence for preventing postoperative sore throat in patients undergoing general anesthesia intubation. It was analyzed from three dimensions: change (change brought by evidence), receiver, and organizational environment (Table 2).

It can be seen from the analysis of the above obstacle factors that evidence needs to be further transformed into a form that is accessible and useable for nurses, such as nursing operation procedures or paths. However, the implementation of some evidence will change the existing procedures, such as preoperative assessment of a patient's throat. The willingness and ability of evidence recipients need to be strengthened and improved, for example, the lack of knowledge and skills related to intubation assessment. Therefore, there is a lack of resources in the organizational environment, especially human resources for anesthesia nurses.

### 2.4. Transformation Strategy of Evidence Transformation

In the process of promoting the clinical transformation of evidence, establishing effective strategies is the guarantee to promote the success of the reform. We should seek available resources and take effective and feasible action plans to promote the success of the change based on understanding the obstacles. A focus group discussion was held to further qualitatively understand the obstacles and promoting factors according to the baseline survey results. Each group consists of 5–9 team members led by a head nurse, and the discussion lasts for 60–120 minutes, which continues until the theoretical arguments are saturated. In the baseline survey, the coincidence rate of 5 review standards in 16 review standards was less than 60%, of which the compliance rate of 2 standards was 0.

As described above, the obstacle factors in the process of evidence transformation are analyzed from three dimensions: change, receiver, and organizational environment, and the change strategy will also aim at these three dimensions.

#### 2.4.1. Strategy of Change Dimension

1. The evaluation list of sore throat prevention after intubation under general anesthesia was determined, printed out, and used through a literature search.
2. I-PARIHS framework helps promote the clinical implementation of research results and guides the analysis of obstacles and promoting factors in the implementation of evidence.
3. Converting the contents and items of measures to prevent sore throat into a flowchart, which is easy to understand and operate.
4. The nursing routine was revised. The content of evaluating intubated patients and the treatment of extubation for intubated patients were written into relevant systems and routines so that the content of the reform was clearly in place in the practice process.
5. Clarifying the links of major changes in the nursing process, such as detailing the medical history of respiratory diseases related to POST and including it in the hospitalization evaluation sheet. Multidisciplinary cooperation is needed to complete the change plan. Unifying evaluation methods and tools. Strengthening the work habits of accurate intubation pipe diameters and operation of each link.

#### 2.4.2. Change Strategy of the Receiver Dimension

1. Enhancing the recipient's willingness to change: it was found that nurses expressed their desire to do something for patients through the investigation, but they had no guidance and did not know how to do it. With these schemes, they could guide nursing work. In order to promote the health of patients, the nursing team retained nurses with relevant health education majors to guide patients and their families; holding a mobilization meeting to allow core personnel such as the director of anesthesiology to support the relevant personnel involved in the practice; any good outcome and the importance of bagging management in practice are important factors to enhance the willingness to change.
2. Enhancing the receiver's knowledge and skills: adopting various forms of training, such as lectures, medical record explanations, watching videos, reading educational manuals, and sputum suction maps; strengthening the training and assessment of nurses and interns in intubation, sputum suction, extubation, and POST safety awareness; strengthening the training of anesthesiologists on the timing, methods, and tools of cuff pressure measurement.
3. Empowerment: the visiting class will assess the POST risk of patients with general anesthesia one day before operation; strengthen the PACU responsibility system and meticulous nursing; and dynamically monitor patients to eliminate the causes of restlessness as soon as possible.
4. Establishing a multidisciplinary team cooperation mechanism: using the Internet such as WeChat to establish communication channels and timely communicate and treat the illness. In-hospital consultation, specialist guidance, and formulation of a POST treatment plan can guarantee the effective implementation of perioperative throat pain care.

#### 2.4.3. Change Strategy of Organizational Environment Dimension

1. The Department of Anesthesiology of our hospital is a training base for regular training and specialized training in Zhenjiang City. It has detailed operating procedures and training methods, which are convenient for training and assessment.
2. Improving the allocation of human nursing resources: there are different forms of propaganda tools in each stage of the perioperative period, and human resources can be adjusted in different links.
3. Formulating the perioperative management path of POST: based on the “Management Pathway for Throat Pain in Patients with Tracheal Intubation under General Anesthesia during Perioperative Period,” evidence was completed, which promoted the pathization of POST management.
4. Optimizing the hospital information system: POST is used as a routine monitoring indicator after general anesthesia and tracheal intubation, and normalized monitoring after extubation and postoperative follow-up is included in the doctor's order system; cuff management standards are formulated and included in surgical quality management information quality control.
5. Using of tools: using ultrasound or CT to measure the diameter of the trachea; applying for a patent for continuous measurement of cuff pressure; PACU is equipped with a system negative pressure gauge; contacting the instrument department to purchase a cuff pressure gauge. Through expert correspondence and evidence-based group discussion, the assessment record sheet for prevention of sore throat in patients with general anesthesia and intubation was jointly revised, including the contents of the recommendations.

### 2.5. The Process of Evidence Implementation

It lasted for 5 months (from June 1, 2020, to October 30, 2020). In June, preparations such as writing health education, nursing manuals, and training nurses were completed before the evidence was implemented. The training content is designed as a small video and courseware, which is placed on the Jingyi teaching platform in the hospital, allowing nurses to participate in the learning, and setting questions for nurses to participate. Evidence-based implementation was implemented from June 1 to October 30, and 192 patients were included.

During the implementation of the evidence, nurses' knowledge of POST prevention was investigated using a questionnaire we designed and compared with the questionnaire in the baseline survey. The questionnaire content was designed based on the best evidence. After the questionnaire was completed, 3 anesthesiologists, 2 evidence-based specialists, and 1 otolaryngologist were consulted. The questionnaire was revised and improved according to expert opinion. The questionnaire consists of 3 parts (dimensions are divided into knowledge, attitude, and behavior). Including 37 questions, each question has a maximum score of 5 points and a minimum score of 1 point, with a total score of 185 points. Questionnaires are sent to nurses through online software. After nurses complete and submit the questionnaires, the system automatically scores the questionnaires. The study found that after the implementation of the evidence, the compliance rate of each item and the score of the questionnaire were improved compared with the baseline survey.

Two graduate students and interns performed data collection according to the review methodology. During the baseline survey and evidence implementation, 5 participants from students studying in the anesthesia operating room participated in data collection. The intern did not know the grouping of patients, and the nurse did not know which patient was performing evidence implementation to avoid the Hawthorne effect. Two graduate students collected the data on the occurrence of POST in patients, and the patient record sheet included general information stating whether POST occurred on admission, and provided admission, operation time, ward, intubation status (intubation size, single-lumen or dual-lumen line), difficult airway, successful extubation, medical information, and equipment involved in POST. To compare the incidence of postoperative POST in intubated patients with general anesthesia after the baseline survey and evidence implementation, patients participating in baseline surveys and evidence implementation should be different.

### 2.6. Statistical Methods

The data were statistically analyzed by SPSS22.0 software, and the counting data were expressed by [*n*(%)]. By using *χ*^2^ test, the VAS score of comfort and the knowledge, belief, and behavior of medical staff were tested by independent sample *T*-test, and the test level *α* = 0.05, with *P* < 0.05 as the difference with statistical significance.

## 3. Results

### 3.1. Structural Dimension System Level

The clinical pathway of intubation for patients under general anesthesia was established (see Figure 1). New technology of selecting suitable endotracheal tube by B-ultrasound to evaluate the tube diameter and setting and monitoring the cuff pressure of endotracheal tube by pressure tester was developed. The follow-up record and quality control book after anesthesia were updated, improving the perioperative throat pain management, endotracheal tube cuff management, postanesthesia visit, and complication management process.

  Step 1: preoperative evaluation to identify high-risk patients with respiratory diseases such as bronchitis and asthma, difficulty airway, and gastrointestinal surgery. In high-risk patients, preventive medication will be given.
  Step 2: intubation management-item preparation: visual intubation equipment, airway nebulizer, ultrasound, tracheal tube, and preventive medication are on standby.
  Step 3: cuff management-airbag pressure filling method: fixed volume injection method, minimum occlusion volume method, minimum lateral leakage test method, dynamic assessment of cuff pressure: 25–30 cm H_2_O, evaluation timing: after tracheal intubation, after a body position change, after pneumoperitoneum, the operation time >6 hours, and after entering the recovery room.
  Step 4: extubation management-sputum suction pressure: 80–100 mmhg; extubation method: a large syringe exhausts the cuff contents and gently removes them to reduce extubation injury.
  Step 5: after extubation, the patient's throat pain and other conditions were promptly assessed, and shifts were handed over and recorded.

### 3.2. Process Dimension Practitioner Level

1. Compliance with evidence-based practices of medical staff: a method similar to the status review was used to review the compliance of the review indicators. A total of 16 indicators were reviewed before and after the implementation of evidence. The results are shown in Figure 2.
2. The score of knowledge-belief-action evaluation of medical staff on the management of intubation prevention for sore throat in patients with general anesthesia: the biggest impact of evidence in the process of clinical translation is the change of practitioners' knowledge, attitude, and behavior (see Table 3).

### 3.3. Outcome Dimension Patient Level

#### 3.3.1. Before and after the Implementation of Evidence

Before and after the implementation of evidence, 151 and 192 patients with general anesthesia who met the inclusion and exclusion criteria were obtained, respectively. There was no statistical difference between the two groups in age, gender, lung disease, department, and body position (see Table 4).

#### 3.3.2. By Comparing the Clinical Outcome Indicators of the Two Groups of Patients

By comparing the clinical outcome indicators of the two groups of patients, the incidence of the sore throat under resting state in patients with general anesthesia and intubation before and after the implementation of evidence, the effect of pain on eating and rest, and the patient's comfort were significantly different (*P* < 0.05). However, there was no significant difference in the incidence of the sore throat under swallowing before and after the implementation of the evidence (*P* > 0.05), as shown in Table 5.

## 4. Discussion

Clinically, less attention is paid to the problem of postoperative sore throat in patients with general anesthesia and intubation. In contrast, we pay more attention to surgical patients' recurrence rate and wound pain after treatment. However, the rehabilitation of patients not only is about unilateral surgical treatment but also needs to pay attention to psychological treatment, prevention of postoperative complications, and comprehensive health guidance. Therefore, scientific, standardized, and systematic nursing also plays a very important role [11]. Some studies have also pointed out that traditional surgical care has been unable to meet the development of modern nursing [12]. This study assessed the implementation of evidence to prevent POST in general anesthesia intubated patients and described the evidence implementation process using the i-PARIHS framework. Evidence implementation is a complex and ongoing process. Evidence-based nursing can start from the actual condition of the patient through methods such as analyzing problems and finding evidence, to formulate a targeted evidence-based nursing plan for the patient, which can bring nursing intervention to the entire perioperative period and improve clinical efficacy. It has played an important role in relieving patients' negative emotions and improving clinical satisfaction [13, 14].

### 4.1. Clinical Practice Based on the Best Evidence Can Effectively Improve the Organizational Environment and Quality of Care

In the past 10 years, both researchers and clinical nursing practitioners in the field of evidence-based nursing have been actively committed to promote the clinical translation of research evidence [15]. We mobilized all the resources throughout the evidence implementation process, with the support of the Nursing Department, Section Chief, and Head Nursing. Authorized by the “top-down” leadership, nurses can provide POST nursing training for patients as long as they have undergone systematic training and mastered relevant skill training. The evidence-based nursing practice for patients with general anesthesia and intubation has changed the previous method of selecting the type of tracheal tube based on estimation. Using B-ultrasound to measure the diameter of the tracheal tube, which is more accurate and less traumatic, changed the finger-feeling method to estimate the pressure and adopted a pressure test instrument to set and monitor endotracheal tube cuff pressure. Standardize endotracheal tube model selection, endotracheal tube cuff management, and endotracheal tube extraction, and incorporate them into quality management to ensure behavioral change. We need to pay attention to the patients themselves and then implement the personalized nursing practice in the process of promoting clinical translation. The problem of “evidence-based intervention can be replaced” also suggests that personalized nursing interventions need to be implemented in the process of evidence transformation. Some evidence needs to be based on the patient's situation and cannot be directly applied. Therefore, in the implementation of evidence, we must implement personalized nursing practice.

### 4.2. Clinical Practice Based on the Best Evidence Improves Nurses' Practice Compliance and Cultivates Nurses' Evidence-Based Concept

This study shows that the implementation rate of the 16 review indicators before and after the implementation of evidence has increased significantly. After the implementation of evidence, in addition to the 62.25% in the first review indicator and the 58.28% in the second review indicator, the achieved rate of the 3 indicators has reached 100%, the rest of the achieved rates are above 60%, and nurses' POST-evidence-based compliance has improved. The evidence-based nursing practice of preventing sore throat in patients with general anesthesia intubation allows nursing staff to solve problems based on scientific evidence when they encounter problems and deal with problems at work, rather than solving problems by experience. For the sustainability of practice, we have repeatedly strengthened the concept of nursing staff from the observation records of baseline survey, training, implementation of the program, and re-examination, and trained and guided the content with low scores in the questionnaire, so that nurses can master nursing knowledge and practical skills, and adopted diversified training such as flowcharts, mission knowledge maps, videos, and case discussions. Propaganda and education are the keys to achieving knowledge, belief, and action that helps clinical staff establish risk awareness, understand the impact of postoperative sore throat, and enhance their execution ability later. The results showed that there was a statistically significant difference in the knowledge, belief, and behavior of clinical medical staff before and after the implementation of evidence (*P* < 0.05). The knowledge, attitude, and behavior were significantly improved, which is very beneficial for improving the compliance of nurses' clinical practice and cultivating nurses' evidence-based concept.

### 4.3. Clinical Practice Based on the Best Evidence Can Improve the Self-Management Ability of Patients with General Anesthesia Intubation to Prevent Sore Throat and Reduce the Incidence of Clinical Sore Throat

The results showed that the incidence of pharyngolaryngeal pain in patients undergoing general anesthesia intubation decreased from 41.7% to 28.1% after the evidence-based practice, and the effects of pain on eating and rest were all lower than before, with a statistically significant difference (*P* < 0.05). However, there was no significant difference in the incidence of sore throat in the swallowing state before and after the implementation of evidence (*P* > 0.05). It shows that the implementation of an evidence-based nursing practice scheme can effectively reduce the incidence of sore throat in patients with general anesthesia intubation at rest. In this study, 20 best pieces of evidence were screened out, 16 review indicators were determined, and practical innovation was implemented. Before the implementation of evidence, the nursing management process of POST had not been established in our hospital, and there is a lack of unified and standardized assessment and preventive measures. Therefore, this study focuses on the concept of “prevention first,” aiming to prevent sore throat in patients with general anesthesia and intubation. The best evidence is applied in the aspects of risk assessment of sore throat in patients with general anesthesia, standardized operation of extubation, and personalized management of sore throat prevention, thereby reducing the incidence of postoperative sore throat and improving the comfort of patients. We can change our behavior and improve our self-management ability by listening to lectures, watching videos, and repeatedly strengthening our training.

Evidence-based practice of the best management strategy for sore throat after general anesthesia intubation has formed the nursing process of general anesthesia intubation, improved the nursing quality and practical compliance, cultivating evidence-based concepts, improved self-management ability, reduced the incidence of clinical sore throat, and effectively promoted the continuous quality improvement of sore throat management after general anesthesia intubation. However, this study was only carried out in one hospital. The sample size of nurses who accepted the reform was relatively small due to the limitation of conditions. Most of them were at risk of gender bias, which affected the authority of the results to a certain extent. In the future, the research program should be carried out in multiple hospitals to evaluate the credibility of its effects scientifically.

## 5. Conclusion

In this study, the evidence retrieval, evaluation, and summary of the prevention and management of sore throat in patients with general anesthesia found that the i-PARIHS evidence-based framework effectively implements clinical management strategies.

## Figures and Tables

**Figure 1:** Clinical pathway of intubation for patients under general anesthesia.

**Figure 2:** Achieved rate of review indicators before and after the implementation of evidence.

**Table 1:** Review indicators and review methods based on the i-PARIHS framework.

Serial number	Review indicators	Review methods
1	Before an operation, doctors and nurses should evaluate the basic condition of patients and actively treat them	Check the nursing record sheet
2	During the operation, anesthesiologists should evaluate the high-risk factors affecting postoperative throat pain	Check the anesthesia record sheet and field survey
3	Anesthesiologists should make a comprehensive assessment of patients with difficult airways and follow-up	Check the preoperative evaluation sheet and postoperative visit records
4	Doctors and nurses should pay attention to the comfort and satisfaction of sore throat	Check the nursing record sheet and field survey
5	Select a video laryngoscope to assist with intubation first	Check the anesthesia record sheet and field survey
6	Anesthesiologists should master the measures to reduce postoperative throat pain and choose the most suitable endotracheal tube	Field survey
7	According to the contraindications of patients, magnesium, licorice, diphenhydramine, corticosteroids (dexamethasone, betamethasone), ketamine, lidocaine, etc., are used locally or intravenously	Check the anesthesia record sheet
8	During the operation, according to factors such as time and body position change, timely use of pressure measuring device to regularly monitor the pressure of the cuff to maintain 25–30cmH2O, and it is not allowed to be measured by the finger sensing method	Field survey
9	When suctioning sputum, anesthesiologists should control the negative pressure of sputum suction at 80∼120 mmHg and fully suck it in every time to avoid repeated operation	Field survey
10	Anesthesiology doctors and nurses should exhaust all the gas in the cuff when extubating the trachea, and gently extubate	Field survey
11	Anesthesiology department doctors and nurses should suck sputum according to the situation of sputum	Field survey
12	Pay attention to your movements when suctioning sputum, please be gentle	Field survey
13	For those with sticky sputum, which is inconvenient to attract, fiber-optic bronchoscopy can be used for sputum aspiration	Field survey

**Table 2:** Obstacles and promoters based on the i-PARIHS framework.

Review indicators	Obstacle factors	Promoting factors
Review indicator 1	I: evidence needs to change the process and system	Team members come from various specialties There are information systems that can be optimized
	R: knowledge and skills are not fully mastered	
	C: at present, hospitals lack relevant admission evaluation procedures and methods	

Review indicator 2	I: evidence needs to change the process and system	Hospital consultation can get specialist treatment guidance
	R: there are many diseases, and medical care may not be able to cure them completely	
	C: there are many patients in each ward, so it is impossible to do fine management	

Review indicator 6	I: evidence content is not included in the evaluation system	In each stage of the perioperative period, there are various forms of publicity tools, and in some links, human resources can be adjusted
	R: the workload of nurses in the ward increased, and their compliance was insufficient	
	C: there is no publicity material for the patients evaluated in this way	

Review indicator 8	I: the evidence failed to transform into an acceptable process and form	The Anesthesiology Department of our hospital is a training base with detailed operation procedures and training methods to facilitate training and assessment
	R: anesthesiologists do not fully understand the content of the evidence	
	C: teaching hospitals, with a large number of personnel for training and further education, are difficult to intubate all at once successfully	

Review indicator 9	I: the measures to reduce postoperative sore throat are not specific enough, and some techniques have certain learning curves	Doctors and nurses have realized the importance of cuff management
	R: there is no accurate tracheal diameter working habit, and some links are not finely operated	
	C: there are no catheters of various types that can meet the demand, and there is no cuff management flow standard and process	

Review indicator 10	I: evidence needs to change existing work habits and processes	The description of the medication process in the literature is relatively detailed
	R: medical staff cannot fully grasp the timing of medication	
	C: some medicines cannot be provided	

Review indicator 11	I: the evidence may conflict with the working environment of doctors and nurses	The price of a pressure measuring device is acceptable
	R: the workload of medical evaluation is large, which is influenced by the cooperation of operation, and it also increases the possibility of forgetting	
	C: there are not enough pressure measuring devices	

Review indicator 12	I:——	Fully attract relevant documents and materials
	R: it is difficult for staff to avoid repeated operations	
	C: the negative pressure gauge value is unclear, and the pressure is not allowed	

Review indicator 14	I:——	The medical staff realizes the importance of gently sucking sputum
	R: the understanding of gentleness among the staff is not consistent enough	
	C: there is no specific illustration of the operation	

Review indicator 16	I:——	There are consensus and guidelines for extubation
	R: I am used to using a small syringe to deflate	
	C: when the patient is restless, it is more difficult to gently pull the tube	

**Table 3:** KAP of surgical medical staff before and after implementation of evidence (score, $\bar{x}\pm S$).

	Knowledge	Attitude	Behavior
Before implementation of evidence	58.91 ± 8.18	35.24 ± 4.55	16.57 ± 4.89
After implementation of the evidence	68.14 ± 6.40	41.47 ± 3.52	21.72 ± 3.36
*t*	−10.516	−12.816	−10.267
*P*	<0.001	<0.001	<0.001

**Table 4:** General situation of research objects (*n*(%)).

Project		Before implementation of evidence	After implementation of evidence	*χ* ^*2*^	*P*
		*N* = 151	*N* = 192		
Age	<60 years old	107 (70.9)	149 (77.6)	2.03	0.154
	≥60 years old	44 (29.1)	43 (22.4)		

Gender	Man	56 (37.1)	78 (40.6)	0.445	0.505
	Woman	95 (62.9)	114 (59.4)		

Dept.	Gastrointestinal surgery	31 (20.5)	43 (22.4)	1.618	0.806
	Chest surgery	27 (17.9)	35 (18.2)		
	Gynecology	33 (21.9)	36 (18.8)		
	Urology	31 (20.5)	39 (20.3)		
	Spine 1	29 (19.2)	39 (20.3)		

Posture	Supine position	45 (29.8)	44 (22.9)	2.762	0.430
	Lateral position	37 (24.5)	52 (27.1)		
	Stone cutting position	34 (22.5)	48 (25.0)		
	Prone position	35 (23.2)	48 (25.0)		

Lung disease	Have	10 (6.6)	17 (8.9)	0.58	0.446
	Without	141 (93.4)	175 (91.1)		

**Table 5:** Comparison of incidence and comfort of the sore throat before and after implementation of evidence (*n*(%)).

Time	Case number	Sore throat at rest	Sore throat in swallowing state	Effect of pain on eating	Effect of pain on rest	Comfort level
Before implementation of evidence	151	63 (41.7)	36 (23.8)	53 (35.1)	52 (34.4)	5.83 (1,10)
After implementation of evidence	192	54 (28.1)	37 (19.3)	20 (10.4)	13 (6.8)	6.65 (0,10)
*χ* ^*2*^ */Z*		6.953(1)	1.183(1)	30.738(1)	42.123(1)	19.955(2)
*P*		<0.05	>0.05	<0.05	<0.05	<0.05

Note: (1) is *χ*^2^ value; (2) is the *z* value.

## Data Availability

No data were used to support this study.

## References

[1] Fai L., Yu-Cih L., Hsiao-Chien T., Chen T. L., Tam K. W., Chen CY. (2015). Effect of Intracuff lidocaine on postoperative sore throat and the Emergence Phenomenon: a systematic review and meta-analysis of Randomized controlled Trials. *PLoS One*.

[2] Sumathi P. A., Shenoy T., Ambareesha M., Krishna H. M. (2008). Controlled comparison between betamethasone gel and lidocaine jelly applied over tracheal tube to reduce postoperative sore throat, cough, and hoarseness of voice. *British Journal of Anaesthesia*.

[3] Maruyama K., Sakai H., Miyazawa H. (2004). Sore throat and hoarseness after total intravenous anaesthesia. *British Journal of Anaesthesia*.

[4] Rajan S., Malayil G., Varghese R., Kumar L. (2017). Comparison of usefulness of ketamine and magnesium sulfate nebulizations for attenuating postoperative sore throat, hoarseness of voice, and cough. *Anesthesia: Essays and Researches*.

[5] An J., Deng X. (2018). Prevention and treatment of sore throat after tracheal intubation. *Medical Review*.

[6] Kuriyama A., Maeda H., Sun R., Aga M. (2018). Topical application of corticosteroids to tracheal tubes to prevent postoperative sore throat in adults undergoing tracheal intubation: a systematic review and meta-analysis. *Anaesthesia*.

[7] Biro P., Seifert B., Pasch T. (2005). Complaints of sore throat after tracheal intubation. *European Journal of Anaesthesiology*.

[8] Huang D., Zhou B., Xiao F., Tang B. (2017). The effect of dexmedetomidine paravertebral nerve block on stress response of patients undergoing thoracotomy. *China Journal of modern medicine*.

[9] Wu W., Bi X., Song L., Liu Z., Zhang J., Huang X. (2016). Application value of Wadian drinking water test in patients with dysphagia after acute stroke. *Journal of Shanghai Jiaotong University*.

[10] Chen S., Chen L., Ye G. (2017). Oxycodone combined with intercostal nerve block for postoperative analgesia after thoracoscopic lobectomy. *China Journal of Modern Medicine*.

[11] Zhang R. (2020). Influence of perioperative evidence-based nursing on complications of patients undergoing thoracic surgery. *Guide of China Medicine*.

[12] Li Y., Jia Y., Li L. (2019). Effect of evidence-based nursing on patients undergoing laparoscopic hysteromyoma surgery. *Electronic Journal of Practical Clinical Nursing*.

[13] Zhang Y., Chen T., Jin M., Gao Y., Hui C., Ren Z. (2017). Evidence-based nursing program to guide perioperative nursing effect of patients with coronary heart disease undergoing interventional diagnosis and treatment. *Journal of Clinical Medicine in Practice*.

[14] Geldenhuys M. J., Downing C. (2020). Evidence-based nursing care for Spinal nursing Immobilization: a systematic review. *Journal of Emergency Nursing*.

[15] Zhou Y., Hu Y., Xing W., Gu Y., Zhu Z. (2018). Design and implementation of evidence transformation and clinical application training program. *Journal of nursing science*.

